# Traditional Chinese Sports under China's Health Strategy

**DOI:** 10.1155/2022/1381464

**Published:** 2022-08-31

**Authors:** Fangyan Yang, Jisheng Zhang

**Affiliations:** ^1^School of Sports and Health, Changsha Medical University, Changsha, Hunan 410219, China; ^2^Adamson University, Manilla, Philippines; ^3^School of Physical Education, Hunan Normal University, Changsha, Hunan 410081, China

## Abstract

Chinese traditional sports are diverse and have rich national cultural connotations. However, with the development of China's Health Strategy, modern sports such as badminton and basketball occupy most of the people's time. On the contrary, there is much less exercise for traditional Chinese sports. Therefore, this paper aims to study Chinese traditional sports under China's Health Strategy and explore its cultural soft power. In this study, participants of all ages in different regions were selected for survey research. Combined with the survey results, the soft power index model of Chinese traditional sports culture is designed. The experimental results showed that for Chinese traditional cultural projects, the cultural soft power index of chui wan was the lowest at 0.568, and the highest was 0.982 in the dragon boat culture soft power index. For each evaluation index, the cultural cognition and cultural attractiveness of Chinese traditional sports were high, but the cultural behavioral power was low. This shows that the soft power model of Chinese traditional sports culture based on the healthy China strategic environment can effectively evaluate the development of traditional Chinese sports, which also can provide suggestions for the development and inheritance of traditional Chinese sports.

## 1. Introduction

Chinese traditional sports are sports activities with national culture that have been formed for thousands of years. Although many sports are learned and understood by not many people, they are not understood by everyone. But sports like dragon boat, lion dance, martial arts, and other well-known sports have brought a lot of health and wellness to the Chinese people. Therefore, under the prosperous situation of modern sports, people must not forget the traditional sports culture, such as chui wan, which is similar to modern golf. chui wan gradually fell into oblivion, while golf developed into a more popular sport in modern times. This is what people must pay attention to China's Health Strategy is crucial to the development goal of national health, as well as to the traditional culture of the nation. However, current China's Health Strategy pays more attention to the improvement of human quality through physical exercise and does not pay much attention to the inheritance and development of traditional sports. If people do not stop the decline of traditional sports, there will be fewer and fewer young people, who can know traditional sports, and fewer and fewer young people can understand their connotations of them. In the end, traditional national sports will be lost or changed.

Traditional sports represent national culture, and many scholars have conducted research on different traditional sports. Liu A attached great importance to the safety of ethnic traditional sports equipment. He believed that the safety of ethnic traditional sports equipment is one of the basic conditions for the development of ethnic traditional sports [1]. Pei and Gong studied the cultural inheritance of traditional sports under the circumstances of social transformation [2]. Ming explored the dissemination mode of national traditional sports culture, so as to obtain an effective dissemination channel, providing a reference for the widespread dissemination of national traditional sports culture [3]. Kogiso's research found that the recognition of traditional and indigenous sports as intangible cultural heritage helps to understand the ambiguity and ambiguity of the sport relative to other cultures [4]. Rogers et al. conducted a heritage study on the local sports culture. He used the new thing of e-sports to combine with traditional sports to achieve the purpose of inheriting sports culture [5]. However, most of the research on traditional sports is limited to the inheritance and development of sports and has not been combined with the background of the current era.

In view of current China's Health Strategy, many scholars have conducted research on it. In order to promote the development of national traditional sports, Pan et al. designed a national traditional sports video distribution system with the help of a software-defined network and mobile edge computing technology combined with the characteristics of China's Health Strategy [6]. Based on the characteristics of China's Health Strategy, Liu et al. assessed and measured the risks of the modernization of traditional sports culture by using the methods of literature, interviews, and simulation experiments [7]. Nölleke and Birkner analyzed the psychological pressure of athletes in the context of current China's Health Strategy [8]. Summerley conducted research on the development of the sports system, focusing on the analysis of the system characteristics under current China's Health Strategy [9]. However, the relevant research is too extensive. No analysis has been carried out for specific sports, and the strategies proposed are not specific enough.

In response to this, this paper combines traditional Chinese sports under China's Health Strategy, adopting a questionnaire survey method. This paper also selects wushu, lion dance, archery, chui wan, diabolo, polo, dragon boat, and cuju, which are eight Chinese traditional sports, to analyze the current situation and development. Aiming at the traditional cultural soft power of sports, the modeling analysis is carried out, in order to rationally analyze the development of the current Chinese traditional sports events. Finally, suggestions for the development of Chinese traditional sports culture based on the weaknesses are given.

## 2. Status Quo of Chinese Traditional Sports under China's Health Strategy

Traditional sports: At present, Chinese scholars focus on qualitative research on strategies, countermeasures, and paths in the international communication of traditional sports, lacking empirical quantitative research. Traditional sports have a long history in China. The construction of this index system starts from the microscopic “audience-effect” type of soft power of traditional sports culture, and systematically and comprehensively introduces new theories, perspectives, and methods into the field of international communication of traditional sports, which focuses on the measurement and evaluation of traditional sports international communication and in-depth research on field evidence [10, 11]. The research on this index evaluation system is helpful for the transformation of traditional sports international communication research from “going out” strategy research to “going in” in-depth research. It is also helpful to improve the effectiveness of the international communication of traditional sports, thereby improving the soft power of traditional sports culture. Some traditional sports are shown in Figure 1.

### 2.1. Traditional Chinese Sports under China's Health Strategy

In the context of China's Health Strategy, the relationship between healthy China and traditional sports is shown in Figure 2. The research on the construction of the index system of the soft power of traditional sports culture cannot only deepen the theoretical cognition of the international communication of traditional sports but also test the communication effect of Chinese traditional sports to the outside world. It is an evaluation of the soft power of Chinese traditional sports culture [12]. The research on the soft power index system of traditional sports culture provides theoretical reference and data support for the international development strategy of traditional sports and “the entry of traditional sports into the Olympics.” Moreover, it can provide a reference for the international development of other Chinese traditional cultures, so as to more effectively implement China's “culture going out” strategy. It can promote the prosperity of Chinese culture on the world cultural stage, enhance the cultural soft power of traditional sports, and enhance the image of traditional sports.

### 2.2. Entropy Weight Method

In establishing the soft power model of traditional sports culture under the healthy China strategy, the first thing to do is to establish the index system. In establishing the index system, it is important to analyze the weight of the index. The larger weight ratio has a greater impact on the model, while the smaller weight ratio has less relationship with the model. Therefore, establishing the weight is to analyze the specific situation of the factors influencing the soft power of traditional sports culture. However, the traditional linear weight calculation method cannot adapt to the diversity of indicators in this paper, so this paper uses the entropy weight method to calculate the weight of indicators.

In this paper, the entropy weight method is used to calculate the weight of each indicator. Entropy originally belonged to the knowledge of thermodynamics and was later introduced into information theory. In the scope of information theory, the functions of information and entropy are to measure the order and uncertainty of a system, respectively. The calculated results of the two have opposite signs and equal absolute values. Information reflects the variability of indicators. The higher the variability of an indicator among all indicators, the more information an indicator provides. In summary, the entropy value is inversely proportional to the weight [13, 14]. When the entropy value of the indicator is small, the weight is heavy. When the entropy value is large, the weight is small. The specific calculation steps are as follows:

Assuming that the evaluation of the soft power of traditional Chinese sports culture is *x*, the first-level index is *I*1, *I*2, *I*3,…, *I*8. The second-level index is *I*_11_,…, *I*_18_,…, *I*_81_,…, *I*_88_, and *S*_*i*_ represents the mean value of the evaluation score of *I*_*i*_. The scores of the importance of each index from 1 to 5 are, respectively, set as five evaluation categories: *C*1, *C*2, *C*3, *C*4, and *C*5. The number of evaluation scores for each index under the second-level index *I*_*ij*_ is *x*_*ij*_1. The *x*_*ij*_1 in proportion of the number of people in the *C*1 evaluation class to the total number of people is set to be *P*(*x*_*ij*_1). If *x*_*ij*_1 is 0, the segment score is not included in the calculation, and *n* is the number of segments included in the calculation as shown in

(1) $$\begin{array}{c} P\left(Xi_{jl}\right)=\frac{Xi_{jl}}{\sum_{l=1}^{5}Xi_{jl}}. \end{array}$$

The entropy value of the soft power evaluation index of Chinese traditional sports culture can be expressed as

(2) $$\begin{array}{c} H\left(X_{ij}\right)=-K\sum_{l=1}^{n}P\left(X_{ijl}\right)\ln\;P\left(X_{ijl}\right). \end{array}$$

Supposing *K*=1/ln  *n*, 0 ≤ *H*(*X*_*ijl*_) ≤ 1 can be satisfied. (1 − *H*(*X*_*ijl*_)) is assumed to be the degree of deviation of *H*(*X*_*ijl*_). Then the entropy weight of *X*_*ijl*_ is as

(3) $$\begin{array}{c} W_{ij}=\frac{\left(1-H\left(X_{ij}\right)\right)}{\sum_{k=1}^{m}\left(1-H\left(X_{ij}\right)\right)}, \end{array}$$

where 0 ≤ *W*_*ij*_ ≤ 1, ∑_*k*=1_^*m*^*W*_*ij*_=1 can also be satisfied.

Among them, *m* is the number of indicators included in the second-level indicator *I*_*i*_, and the score of the first-level indicator is the sum of the average score of the second-level indicator multiplied by the entropy weight as shown in

(4) $$\begin{array}{c} S_{i}=\sum_{k=1}^{m}W_{ij}*S_{ij}. \end{array}$$

From the entropy value 1 and entropy weight 2 of each index, the entropy value and entropy weight of each index is calculated as

(5) $$\begin{array}{c} H\left(X_{i}\right)=\sum_{k=1}^{m}W_{ij}H\left(X_{ij}\right), \end{array}$$

(6) $$\begin{array}{c} W_{i}=\left(\frac{1-H\left(X_{i}\right)}{\sum_{k=1}^{m}W_{ij}H\left(X_{i}\right)}\right), \end{array}$$

(7) $$\begin{array}{c} S_{i}=\sum_{k=1}^{m}W_{ij}*S_{ij}. \end{array}$$

The comprehensive entropy weight of the soft power evaluation index of Chinese traditional sports culture can be expressed as

(8) $$\begin{array}{c} W_{ij}=w_{ij}*w_{i}. \end{array}$$

The importance of each layer of indicators is the final entropy weight, which is the weight in the soft power evaluation of Chinese traditional sports culture [15].

## 3. Construction of the Comprehensive Index of Soft Power of Chinese Traditional Sports Culture

### 3.1. Indicator Construction

The construction of the indicator system and the selection of specific indicators are complex tasks. The designer of the index system is required to have a very clear understanding of the evaluation object, evaluation content, and evaluation purpose, as well as a certain depth and breadth of relevant basic theories.

The evaluation index system of traditional sports culture soft power adopts the method of combining theory first and practice correction. First of all, guided by the evaluation goal, based on the “three-layer theory” of traditional sports culture, audience theory, communication effect theory, and cultural soft power theory, the theoretical model of traditional sports culture soft power is constructed. Then, on the basis of the theoretical model, specific evaluation indicators are selected for pretesting [16, 17]. The research on the construction of the index system in this paper is difficult to determine the importance and practicability of the index by using the Delphi method for multiple rounds of scoring.

For whether an evaluation system is scientific and reasonable, in addition to scientifically constructing a reasonable theoretical framework, it is crucial to select specific key indicators according to the evaluation object and evaluation purpose. The selection process of specific indicators is the same process as the selection process of the survey items of the questionnaire. It is established through expert interviews and reliability tests combined with theoretical models [18].

### 3.2. Indicator Establishment

Combined with the previous research on cultural soft power, the evaluation index system of traditional sports culture soft power is composed of a four-level comprehensive evaluation index system, that is, 1 target layer, 3 first-level indicators, 9 second-level indicators, 29 third-level indicators, and 200 measurement items. The first-level indicators include traditional sports culture cognition, traditional cultural attractiveness, and traditional sports cultural behavior. The specific indicators are as follows:

The cognition of traditional sports culture, which is a measure of the foreign audience's cognition of all elements of Chinese traditional sports culture and a first-level qualitative index for evaluating the soft power of traditional sports culture, includes three secondary indicators: the cognition of traditional sports material culture, the cultural cognition of traditional sports system, and the cultural cognition of traditional sports spirit. The three second-level indicators include a total of 10 third-level indicators. The traditional sports material and cultural cognition include four third-level indicators (traditional sports equipment cognition, traditional sports landscape cognition, traditional sports boxing cognition, and traditional sports celebrity cognition). The cultural cognition of the traditional sports system includes four three-level indicators (traditional ritual cognition, organizational cognition, traditional sports event cognition, and traditional sports ethics cognition). The cultural cognitive ability of traditional sports spirit includes two three-level indicators (the cognitive ability of traditional sports thinking concept and the cultural cognitive ability of traditional sports art).

The attractiveness of traditional sports culture refers to the measure of the attractiveness of Chinese traditional sports culture to foreign audiences. The attractiveness of traditional sports culture is mainly measured from the perspective of the audience to measure the conceptual recognition and emotional love or interest of foreign audiences in the various elements of Chinese traditional sports culture. It is a first-level indicator for evaluating the soft power of traditional sports culture, including three second-level indicators: the material cultural attraction of traditional sports, the cultural attraction of traditional sports system, and the cultural attraction of traditional sports spirit. The three second-level indicators include a total of 10 third-level indicators. The physical and cultural attraction of traditional sports includes four three-level indicators (attraction of traditional sports equipment, attraction of traditional sports landscape, attraction of traditional sports boxing, and attraction of traditional sports celebrities). The cultural attraction of the traditional sports system includes four three-level indicators (the attraction of traditional rituals, the attraction of organizational institutions, the attraction of traditional sports events, and the attraction of traditional sports ethics). The cultural attractiveness of traditional sports spirit includes two three-level indicators (the attractiveness of traditional sports thinking concepts and the cultural attractiveness of traditional sports arts).

The traditional sports culture behavior force measures the traditional sports behavior of foreign audiences. Traditional sports culture behavioral power mainly measures the use of foreign audiences' use of Chinese traditional sports culture communication channels and the practice of audience behavior from the perspective of audiences. It is the first-level evaluation index of traditional sports culture's soft power. It includes three secondary indicators, namely traditional sports information contact behavior, traditional sports technical practice behavior, and traditional sports culture consumption behavior. The three second-level indicators include a total of 11 third-level indicators. The traditional sports information contact behavior includes four three-level indicators (the number of traditional sports information contacts, the contact time of traditional sports information, the number of traditional media types, and the number of network new media types). The traditional sports technique practice behavior includes three three-level indicators (the number of traditional sports boxing exercises, the number of traditional sports weekly training, and the traditional sports technique practice time). The consumption behavior of traditional sports culture includes four three-level indicators (the number of traditional sports books purchased, the number of traditional sports craft souvenirs purchased, the number of traditional sports clothing and equipment purchased, and the number of traditional sports film and television performances purchased).

### 3.3. Indicator Internal Consistency Reliability Test

Internal consistency reliability, also known as homogeneity reliability, refers to the degree of consistency between the indicators of the indicator system (among all items within the scale). The internal consistency reliability coefficient mainly reflects the correlation between various indicators (each measurement item). Internal consistency has two meanings. One is that all items measure the same concept or psychological trait. The other is that all item scores have a high positive correlation [19, 20].

The calculation methods of internal consistency reliability include split-half reliability, Cronbach's Alpha, and Hoyt reliability. This paper mainly uses the Cronbach's *α* coefficient (Cronbach's Alpha), which is the most common way to assess the internal consistency of a model or various items in a survey.

In the field of social science research, each scale often contains multiple dimensions or levels, and each dimension is measured by multiple subscales. Therefore, in addition to providing the reliability coefficients of the total scale, users should also provide the reliability coefficients of each subscale. The closer the internal consistency reliability coefficient is to 1, the higher the internal consistency between each index (each measurement item) will be. The internal consistency reliability evaluation criteria are shown in Table 1.

As shown in Table 2, the Cronbach's *α* coefficient of the total index of traditional sports culture soft power is 0.782. According to the internal consistency reliability evaluation standard, it is acceptable, indicating that the internal consistency of the sub indicators at all levels of the total index is acceptable. The Cronbach coefficients of the three first-level indicators of traditional sports culture soft power: *A*—traditional sports culture cognition, *B*—traditional sports culture attractiveness, and *C*—traditional sports culture behavioral power are 0.799, 0.921, and 0.734, respectively. According to the internal consistency reliability evaluation standard, the internal consistency of *B*'s traditional sports culture attractiveness is much better than the internal consistency of *A*'s traditional sports culture's cognitive ability and *B*'s traditional sports culture's behavioral ability, and the consistency of behavioral ability is relatively the worst.

As shown in Table 3, in the internal consistency reliability test of the secondary indicators, *A*1 traditional sports material cultural cognition, *B*1 traditional sports material cultural attraction, *B*2 traditional sports institutional cultural attraction, and *C*3 traditional sports culture consumption behavior Cronbach's alpha coefficients are all above 0.70 (They are 0.798, 0.931, 0.718, and 0.753, respectively). It shows that the internal consistency is high. The Cronbach's *α* coefficient of the secondary index *B*3 traditional sports spirit and cultural attraction is 0.690, and its internal consistency is also good according to the internal consistency reliability evaluation standard. However, the Cronbach *α* coefficients of the secondary indicators *A*2 traditional sports system cultural cognition, *A*3 traditional sports spirit cultural cognition, *C*1 traditional sports information contact behavior, and *C*2 traditional sports practice behavior are 0.548, 0.539, 0.579, and 0.599, respectively. According to the internal consistency reliability evaluation standard, when 0.50≤ Cronbach's *α* coefficient <0.60, it is unacceptable and needs to be modified appropriately.

Judging from the Cronbach coefficients of the three-level indicators, only the cognitive ability of *A*21 traditional rituals, the cognitive ability of *A*31 traditional sports thinking concepts, and the attractiveness of *B*21 traditional rituals are lower, but they are all greater than 0.50. Internal consistency is acceptable. The rest are higher than 0.80 or 0.90, and the degree of internal consistency is ideal or very ideal.

## 4. Analysis of the Soft Power Model of Chinese Traditional Sports Culture

### 4.1. Cultural Cognition Index Results and Deconstruction

The cultural cognition of traditional sports includes material cultural cognition, institutional cultural cognition, and spiritual cultural cognition. Among them, the cognitive ability of traditional sports material culture is composed of four three-level indicators: *A*11—traditional sports equipment cognition, *A*12—traditional sports landscape cognition, *A*13—traditional sports boxing cognition, and *A*14—traditional sports celebrity cognition. The cultural cognition of the traditional sports system is composed of three three-level indicators: *A*21—traditional ritual cognition, *A*22—organization event cognition, and *A*23—traditional sports moral cognition. The cultural cognitive ability of traditional sports spirit is composed of two three-level indicators—*A*31, traditional sports thinking concept cognitive ability and *A*32, traditional sports art cultural cognitive ability. After calculating the weights, the scores of the eight traditional sports in each index of traditional sports spirit and cultural cognition are shown in Figure 3.

The results in Figure show that, in terms of each index, the cognitive ability of traditional sports equipment and traditional sports celebrities (except chui wan) scored relatively high among the respondents. As far as traditional sports are concerned, archery had relatively high scores in various indicators of cognition in traditional sports landscapes, and the lowest score was chui wan. Among all the respondents and all indicators, the cognition of traditional sports celebrities was the lowest among those surveyed in chui wan.

As shown in Figure 3(b), in terms of each index, among the three three-level indicators of traditional sports material culture cognition, traditional ritual cognition and traditional sports moral cognition were relatively high. As far as traditional sports were concerned, archery respondents were relatively high in all three indicators, while chui wan was relatively low. Among all the respondents and all indicators, the respondents of diabolo had the highest awareness of traditional sports ethics, and the respondents of chui wan had the lowest awareness of organizing events.

As shown in Figure 3(c), among the two three-level indicators of traditional sports spirit and cultural cognition, the cognition of traditional sports thinking concepts was relatively high. As far as traditional sports were concerned, archery respondents were relatively high in both indicators, while hammering was relatively low. Among all the respondents and all the indicators, the respondents of diabolo had the highest cognitive ability of traditional sports thinking concepts, and the respondents of chui wan had the lowest cognitive ability of traditional sports thinking concepts.

### 4.2. Cultural Attractiveness Index Results and Deconstruction

The first-level indicator of the soft power of traditional sports culture, the attractiveness of traditional sports culture, is composed of three second-level indicators: the material cultural attraction of traditional sports, the cultural attraction of traditional sports system, and the spiritual-cultural attraction of traditional sports. The detailed indicators are as follows: The physical and cultural attraction of traditional sports is composed of four three-level indicators—*B*11, traditional sports equipment attraction, *B*12, traditional sports landscape attraction, *B*13, traditional sports boxing attraction, and *A*14, traditional sports celebrity attraction. The cultural attractiveness of the traditional sports system is composed of three three-level indicators—*B*21, traditional ritual attraction, *B*22, organized event attraction, and *B*23, traditional sports moral attraction. The cultural attraction of traditional sports spirit is composed of two three-level indicators, *B*31, traditional sports ideological and conceptual attraction and *B*32, traditional sports art, and cultural attraction. After calculating the weights, the scores of the eight traditional sports in various indicators of traditional sports spirit and cultural attractiveness are shown in Figure 4.

As shown in Figure 4(a), in terms of the four indicators of traditional sports material cultural attractiveness, traditional sports celebrity attraction scored relatively high among respondents in each traditional sports event. As far as traditional sports were concerned, dragon boat had relatively low attractiveness in traditional sports landscapes and traditional sports, while diabolo had the highest attraction in traditional sports celebrities.

As shown in Figure 4(b), in terms of the cultural attractiveness index of the traditional sports system, the traditional sports' moral attractiveness scored relatively high among the respondents of various traditional sports. As far as traditional sports were concerned, the respondents of diabolo were relatively high in all indicators.

As shown in Figure 4(c), in terms of the cultural attractiveness of traditionall sports spirit, the scores of respondents in traditional sports thinking and concept attractiveness were relatively high. As far as traditional sports were concerned, the respondents of diabolo were relatively high in all indicators.

### 4.3. Cultural Behavior Index Results and Deconstruction

The first-level index of traditional cultural behavior is composed of three second-level indicators: traditional sports information contact behavior, traditional sports practice behavior, and traditional sports culture consumption behavior. Details are as follows:

The second-level indicator of traditional sports information contact behavior is composed of four third-level indicators: *C*11—the number of traditional sports information contacts, *C*12—the contact time of traditional sports information, *C*13—the types of traditional sports information contact channels, and *C*14—the types of traditional sports information contact channels. The second-level index of traditional sports technology practice behavior is composed of three third-level indicators: *C*21—the number of traditional sports boxing exercises, *C*22—the number of traditional sports weekly training, and *C*23—traditional sports training time. The second-level indicators of traditional sports culture consumption behavior include four three-level indicators: *C*31—the number of books purchased on traditional sports, *C*32—the number of traditional sports craftsmanship, the number of souvenirs purchased, *C*33—the number of traditional sports clothing and equipment purchased, and *C*34—the number of purchases of traditional sports films and performances. After calculating the weights, the scores of the eight traditional sports culture items in various indicators of traditional sports culture consumption behavior are shown in Figure 5.

As shown in Figure 5(a), the scores of various indicators of traditional sports information contact behavior were relatively low, and the average monthly number of traditional sports information contacts was relatively high among the respondents of various traditional sports items. In terms of traditional sports, archery and diabolo scored relatively high in various indicators. In terms of comparison of all indicators of traditional sports respondents, the number of new media types of the respondents in chui wan was the lowest.

As shown in Figure 5(b), among the various indicators of traditional sports technique practice behavior, the scores of respondents in traditional sports training time were relatively high, and the scores of traditional sports boxing were relatively low. There was little difference in the scores of the three indicators among the respondents who practice traditional sports in various traditional sports.

As shown in Figure 5(c), in terms of the four indicators of traditional sports culture consumption behavior, the number of purchases of traditional sports films and performances was the highest, and the number of traditional sports books purchased was the lowest. As far as traditional sports were concerned, archery and diabolo were relatively high, and the indicators of hammering were relatively low.

## 5. Conclusion

This paper adopts the idea of combining theory and practice to construct the evaluation index system of traditional sports culture soft power and uses the objective weighting method to determine the index weight coefficient. Finally, this article constructs a comprehensive evaluation index system of traditional sports culture soft power. Among the weight coefficients of the three first-level indicators in the soft power evaluation index system of traditional sports culture, the weight coefficient of traditional sports culture attraction is the highest (0.3793). The weight coefficient of traditional sports culture behavioral ability is the second (0.3473), and the weight coefficient of traditional sports culture cognitive ability is the lowest (0.2734). This shows that the soft power of traditional sports culture is more susceptible to the influence of attractiveness and behavioral indicators, and it also reflects that more attention should be paid to the attractiveness and behavioral indicators when implementing strategic countermeasures to improve the soft power of traditional sports culture. Although the research in this paper has achieved relatively satisfactory results, there are still some shortcomings, such as the low reliability of some indicators of cultural cognition and cultural attractiveness. Therefore, in the follow-up research, the selection of indicators will be optimized to make the cultural soft power model more realistic.

## Figures and Tables

**Figure 1:** Traditional sports.

**Figure 2:** Healthy China and traditional sports.

**Figure 3:** Analysis of the weight of traditional sports culture cognitive power. (a) Material cultural cognition. (b) Institutional cultural cognition. (c) Spiritual cultural cognition.

**Figure 4:** Analysis of the weight of traditional sports culture attraction. (a) Material cultural attraction. (b) Institutional cultural attraction. (c) Spiritual cultural attraction.

**Figure 5:** Analysis of the weight of traditional sports culture behavioral power. (a) Information contact behavior. (b) Practice behavior. (c) Cultural consumption attractiveness.

**Table 1:** Internal consistency reliability coefficient evaluation standard table.

	Total amount table	Component table
*α* < 0.6	Not ideal, give up	Not ideal, give up
0.6 ≤ *α* < 0.8	Grudgingly accept	Grudgingly accept
0.8 ≤ *α* < 0.9	Accepted, with high confidence	Accepted, with high confidence
*α* ≥ 0.9	Very ideal	Very ideal

**Table 2:** Total scale and primary indicator Cronbach's alpha.

Index	Index number	Cronbach's alpha
Total index	29	0.801
*A* cultural cognition	9	0.798
*B* cultural attraction	9	0.931
*C* cultural behavior	11	0.719

**Table 3:** Secondary indicator Cronbach's alpha.

Index	Index number	Cronbach's alpha
*A*1 material and cultural cognition	4	0.689
*A*2 institutional cultural cognition	3	0.891
*A*3 mental and cultural cognition	2	0.76
*B*1 material and cultural attraction	4	0.671
*B*2 institutional cultural attraction	3	0.711
*B*3 spiritual and cultural attraction	2	0.787
*C*1 information contact behavior	4	0.664
*C*2 practice behavior	3	0.676
*C*3 cultural consumption behavior	4	0.841

## Data Availability

The data used to support the findings of this study are available from the corresponding author upon request.
